The article "Screening of potential biomarkers for polycystic ovary syndrome and identification of expression and immune characteristics" was retracted in 2025. Reasons: unreliable results or conclusions; concerns about the methods.

# Screening of potential biomarkers for polycystic ovary syndrome and identification of expression and immune characteristics

**DOI:** 10.1371/journal.pone.0293447

**Published:** 2023-10-26

**Authors:** Shuang Liu, Xuanpeng Zhao, Qingyan Meng, Baoshan Li

**Affiliations:** The Reproductive Laboratory, Shenyang Jinghua Hospital, Shenyang, China; Xiangya Hospital Central South University, CHINA

## Abstract

**Background:**

Polycystic ovary syndrome (PCOS) seriously affects the fertility and health of women of childbearing age. We look forward to finding potential biomarkers for PCOS that can aid clinical diagnosis.

**Methods:**

We acquired PCOS and normal granulosa cell (GC) expression profiles from the Gene Expression Omnibus (GEO) database. After data preprocessing, differentially expressed genes (DEGs) were screened by limma package, and Gene Ontology (GO) and Kyoto Encyclopedia of Genes and Genomes (KEGG) enrichment analysis and Gene Set Enrichment Analysis (GSEA) were performed. Recursive feature elimination (RFE) algorithm and the least absolute shrinkage and selection operator (LASSO) Cox regression analysis were used to acquire feature genes as potential biomarkers. Time-dependent receiver operator characteristic curve (ROC curve) and Confusion matrix were used to verify the classification performance of biomarkers. Then, the expression characteristics of biomarkers in PCOS and normal cells were analyzed, and the insulin resistance (IR) score of samples was computed by ssGSEA. Immune characterization of biomarkers was evaluated using MCP counter and single sample gene set enrichment analysis (ssGSEA). Finally, the correlation between biomarkers and the scores of each pathway was assessed.

**Results:**

We acquired 93 DEGs, and the enrichment results indicated that most of DEGs in PCOS group were significantly enriched in immune-related biological pathways. Further screening results indicated that JDP2 and HMOX1 were potential biomarkers. The area under ROC curve (AUC) value and Confusion matrix of the two biomarkers were ideal when separated and combined. In the combination, the training set AUC = 0.929 and the test set AUC = 0.917 indicated good diagnostic performance of the two biomarkers. Both biomarkers were highly expressed in the PCOS group, and both biomarkers, which should be suppressed in the preovulation phase, were elevated in PCOS tissues. The IR score of PCOS group was higher, and the expression of JDP2 and HMOX1 showed a significant positive correlation with IR score. Most immune cell scores and immune infiltration results were significantly higher in PCOS. Comprehensive analysis indicated that the two biomarkers had strong correlation with immune-related pathways.

The article "Screening of potential biomarkers for polycystic ovary syndrome and identification of expression and immune characteristics" was retracted in 2025. Reasons: unreliable results or conclusions; concerns about the methods.

**Conclusion:**

We acquired two potential biomarkers, JDP2 and HMOX1. We found that they were highly expressed in the PCOS and had a strong positive correlation with immune-related pathways.

## 1 Introduction

Polycystic ovary syndrome (PCOS) is a widespread disorder of endocrine and metabolic abnormalities that affects up to 15% of women of adolescent and gestational age [1]. PCOS can lead to abnormalities in the female reproductive system and immune system, and the clinical manifestations are generally irregular menstruation and even amenorrhea, excessive male hormones, polycystic ovary morphology [2]. Severe PCOS can lead to insulin resistance (IR), female anovulatory infertility, pathological obesity, autoimmune diseases, local or whole body inflammation and many other diseases [3, 4]. The specific causes of PCOS are complex and multi-systemic, lack of targeted treatment, different diagnostic criteria and methods, and need to be adjusted according to different clinical symptoms [5]. In addition, it has been shown that follicular excess and increased size of the ovaries in PCOS are associated with insulin resistance (IR) and that the number of follicles may also be a predictor of IR [6]. However, the pathogenesis of PCOS is not yet perfect, and there are many hypotheses about different pathogenesis factors, such as chronic low-grade inflammation, genetic factors, lifestyle, post-translational modification mechanism of PCOS, and ovarian autophagy mechanism [7–9].

Ovarian granulosa cells (GC) are the main constituent cells of follicles, which can divide and differentiate in different degrees with the growth of follicles, and also play an important role in hormone secretion [10]. Abnormalities in GC can lead to ovary-related diseases, such as a deficiency of Rpg5 (an autophagy protein) in GC that can lead to premature ovarian failure [11]. Inflammation caused by high levels of male hormones can also lead to GC pyroptosis, causing ovarian function decline and tissue fibrosis [12]. The abnormal communication of oocyte and follicular cells and the damage of GC may be the key to PCOS, such as the damage of transregional projection in communication [13]. Therefore, understanding the abnormal mechanism of GC is very important for the study of PCOS.

The purpose of this study was to search for potential biomarkers of PCOS and explore the association between biomarkers and immune status in PCOS. In this research, Recursive Feature Elimination (RFE) algorithm was used for selection of feature gene. The prediction strength and practicability of this algorithm are relatively good, and it has been used many times in the screening of biomarkers for different diseases, such as chronic obstructive pulmonary disease, keloid disorder, and triple negative breast cancer [14–16].

The article "Screening of potential biomarkers for polycystic ovary syndrome and identification of expression and immune characteristics" was retracted in 2025. Reasons: unreliable results or conclusions; concerns about the methods.

## 2 Material and methods

### 2.1 Data sources and preprocessing

**(1) Data sources.** Granulosa cell expression profiles of PCOS were acquired from Gene Expression Omnibus (GEO) database: GSE137684, GSE34526, GSE138518, GSE168404, GSE155489 (Table 1) [17]. RNA-Seq expression profiles (GSE107746) of granulosa cells at five follicular development stages were acquired from GEO database.

**Table 1:** Information of datasets.

dataset	Platforms	PCOS	Control	Experiment type
GSE137684	GPL17077	8	4	array
GSE34526	GPL570	7	3	array
GSE138518	GPL11154	3	3	high throughput sequencing
GSE168404	GPL16791	5	5	high throughput sequencing
GSE155489	GPL20795	4	4	high throughput sequencing

**(2) Data preprocessing.** GSE137684 and GSE34526 (microarray) were combined as a training set. GSE138518, GSE168404, and GSE155489 (RNA-Seq) were combined as a test set, and the batch effect was removed using the ComBat function of the sva package (Figure S1) [18]. RNA-Seq expression profiles were converted into TPM format data.

### 2.2 Identification and enrichment of differentially expressed genes (DEGs)

We used limma package to identify DEGs, and the threshold was set to p < 0.05 and | log2FC| > log2(1.5) [19]. Gene Ontology (GO) and Kyoto Encyclopedia of Genes and Genomes (KEGG) analyses were performed on all upregulated DEGs in PCOS using the R software clusterProfiler package to assess their pathway processes [20], biological processes (BP), cellular components (CC), and molecular functions (MF). Gene set enrichment analysis (GSEA) was performed to further assess the enrichment of relevant functional pathways between different groups [21].

### 2.3 Selection and verification of biomarkers

The recursive feature elimination (RFE) algorithm of the caret package is used for characteristic gene selection and 10x cross-validation [22]. The key parameters we chose are: functions = "rfFuncs", method = "cv", number = 10. We then used LASSO regression of the glmnet package for characteristic gene screening [23]. The parameters chosen for the LASSO regression analysis were: nfolds = 5, family = ’binomial’, type. Measure = ’deviance’. The potential biomarkers were acquired by comprehensive analysis of the two algorithms. To further assess the diagnostic performance of candidate biomarkers, the receiver operating characteristic (ROC) curve and its area under the curve (AUC), accuracy, sensitivity, and specificity were computed using the R software timeROC package and confusion matrix [24]. The gene of Insulin secretion pathway was downloaded from KEGG, and the IR score of each sample was computed by ssGSEA method [25].

The article "Screening of potential biomarkers for polycystic ovary syndrome and identification of expression and immune characteristics" was retracted in 2025. Reasons: unreliable results or conclusions; concerns about the methods.

### 2.4 Analysis of immune infiltration and biological pathways

The MCP counter algorithm was used to estimate the relative proportion of 10 kinds of immune cells [26]. MCP counter is an algorithm that allows stable quantification of the absolute abundance of 2 stromal and 8 immune cell populations in heterogeneous tissues from transcriptomic data [27]. The infiltration of 28 immune cells was represented by an enrichment score, which was computed using a single sample gene set enrichment analysis (ssGSEA) of the GSVA package [21]. We acquired the ssGSEA scores of each sample in the HALLMARK Pathway, and computed the correlation between the biomarkers and the scores of each pathway. In addition, we obtained 103 immunomodulation-related genes based on previous studies and evaluated the relationship between PCOS-related genes and these genes using the spearman method [28].

### 2.5 Statistical analysis

The difference between the two groups was tested by Wilcoxon rank sum test [29]. Kruskal-Wallis test was used for the difference between the three groups and more [30]. Correlation analysis was computed using pearson method [31]. The P less than 0.05 is defined as a significant difference. Notably, * means p-value less than 0.05; ** means p-value less than 0.01; *** means p-value less than 0.001, and **** means p-value less than 0.0001. ns means there is no significant difference between two groups.

## 3 Results

### 3.1 Acquisition and enrichment analysis of DEGs

DEGs in PCOS group and normal control group were identified in microarray cohort and RNA-Seq cohort. A total of 1044 up-regulated genes and 695 and down-regulated genes were acquired in the microarray cohort (Fig 1A). A total of 464 up-regulated genes and 103 down-regulated genes were acquired in the RNA-Seq cohort (Fig 1B). Cross analysis between the two cohorts revealed 93 common DEGs (Fig 1C).

**Fig 1:** Acquisition and enrichment analysis of DEGs. A: PCOS data of microarray and DEGs volcano map of control group; B: PCOS data of the RNA-Seq cohort and DEGs volcano map of the control group; C: 93 common differential genes in the two datasets; D: GO and KEGG enrichment analysis of up-regulated genes in all PCOS data.

By KEGG enrichment analysis, Tuberculosis, Epstein-Barr virus infection, Phagosome and other pathway processes were found to be significant. Neutrophil activation, neutrophil activation involved in immune response, neutrophil degranulation, neutrophil mediated immunity is a process with significant enrichment in BP. Secretory granule membrane was the most significantly enriched component in CC. Actin binding and GTPase binding were the two most enriched functions in MF. (Fig 1D). These results suggest that PCOS is primarily associated with immune-related pathways and biological functions in patients. In addition, GSEA analysis indicated that the enriched gene set was closely related to antigen processing and presentation, B cell receptor signaling pathway, and neutrophil-mediated immunity in the PCOS group (Fig 2A and 2C). Metabolism-related pathway activity was significantly higher in the normal control group (Fig 2B).

The article "Screening of potential biomarkers for polycystic ovary syndrome and identification of expression and immune characteristics" was retracted in 2025. Reasons: unreliable results or conclusions; concerns about the methods.

**Fig 2:** GSEA analysis in PCOS group and control group. A, C: GSEA showed immune signaling pathways and biological processes in the PCOS group; B, D: The 5 pathways most associated with the control group.

### 3.2 Screening and validation of biomarkers

RFE and LASSO regression were used to screen 93 differential genes. Three genes were acquired by RFE algorithm: JDP2, HMOX1 and BNIP3 (Fig 3A). Nine genes were acquired by LASSO regression: TP53I11, MXRA8, JDP2, CDH3, STC1, HMOX1, COLQ, LTBP1 and LGMN (Fig 3B and 3C). JDP2 and HMOX1 are the common genes acquired by the two algorithms.

**Fig 3:** Screening and validation of biomarkers. A: Screening biomarkers based on RFE algorithm; B, C: Characteristic gene selection by LASSO regression; D: ROC curve of JDP2 and HMOX1 in training set; E: ROC curve of the training set combination JDP2 and HMOX1; F: Training set model performance evaluation; G: ROC curve of JDP2 and HMOX1 in test set; H: ROC curve of the test set combination JDP2 and HMOX1; I: Test set model performance evaluation.

ROC analysis indicated that JDP2 and HMOX1 were of high value in distinguishing PCOS from normal samples, and the AUC values of the training set and the test set were ideal (Fig 3D and 3G). The ROC curve after the combination of the two genes still had a high AUC value, with the training set AUC = 0.929 and the test set AUC = 0.917(Fig 3E and 3H). Confusion matrix results showed that the Sensitivity of the training set and the test set were both greater than 0.8, and the Accuracy was greater than 0.9. In addition, we demonstrated using PCA analysis that JDP2 and HMOX1 were able to distinguish between PCOS samples and normal samples (S1 Fig). These results indicating that the two biomarkers identified had good classification performance (Fig 3F and 3I).

### 3.3 Analysis of expression of two biomarkers

Next, we explored the differences in the expression of two genes in PCOS and normal controls. In both the training set and the test set, JDP2 and HMOX1 showed high expression in the PCOS group, P < 0.001 (Fig 4A and 4B). At the same time, the specific expression of markers at different developmental stages was explored. Here, their expression in granulosa cells at different follicular development stages was compared by dataset GSE107746. The results indicated that JDP2 and HMOX1, which should be inhibited during the pre-ovulation phase, were elevated in PCOS tissues, suggesting that high levels of JDP2 and HMOX1 expression in granulosa cells may also play an important role in follicular development in PCOS (Fig 4C).

The article "Screening of potential biomarkers for polycystic ovary syndrome and identification of expression and immune characteristics" was retracted in 2025. Reasons: unreliable results or conclusions; concerns about the methods.

**Fig 4:** Analysis of expression of two biomarkers. A: The expression of JDP2 and HMOX1 in the training set; B: The expression of JDP2 and HMOX1 in the test set; C: Expression of JDP2 and HMOX1 in granulosa cells at different follicular development stages; D: The difference of IR score between PCOS and normal control group; E: JDP2 and HMOX1 were correlated with IR scores.

Insulin resistance (IR) plays an important role in the development of PCOS, and the IR score for each sample was computed using the ssGSEA method. The results indicated that PCOS had a higher IR score (Fig 4D). The expressions of JDP2 and HMOX1 showed a significant positive correlation with IR score, and the correlation of HMOX1 was stronger, P = 0.00076 (Fig 4E). These results demonstrate the presence of higher levels of insulin resistance in PCOS patients and that patients with higher IR scores will have high expression of JDP2 and HMOX1.

### 3.4 Relationship of biomarkers to immune infiltration and biological pathways

We compared 28 kinds of immune cell scores between PCOS and normal control samples, and the results indicated that 21 kinds of immune cell scores were significantly higher in PCOS (Fig 5A, S1 Table). The immune infiltration results acquired by MCP Counter algorithm are consistent with the above, and the scores of B lineage, Monocytic lineage, and Neutrophils are higher than those of PCOS (Fig 5B). Correlation analysis was performed to assess the relationship between biomarkers and infiltrating immune cells. JDP2 showed significant positive correlation with T cells and cytotoxic lymphocytes, with P values less than 0.05 (Fig 5C). HMOX1 showed significant positive correlation with monocytes and myeloid dendritic cells. The maximum value of P is 0.036 (Fig 5D). In addition, we further explored the relationship of PCOS-related genes with chemokine-related genes, immunoinhibitor-related genes, immunostimulator-related genes, MHC-related genes and receptor-related genes. As shown in S2 Fig, we found that PCOS-associated genes were significantly associated with most of the immunomodulatory genes, such as CCL4, CXCL17, CSF1R, CD48, IL6R, HLA, CCR1 and CCR5.

**Fig 5:** Association of biomarkers with immune infiltration. A: The immune scores between PCOS and control group were compared by ssGSEA method. B: MCP Counter method was used to compare the immune scores between PCOS and control group. C: The correlation between JDP2 and immune cells; D: Correlation between HMOX1 and immune cells.

The article "Screening of potential biomarkers for polycystic ovary syndrome and identification of expression and immune characteristics" was retracted in 2025. Reasons: unreliable results or conclusions; concerns about the methods.

We computed the ssGSEA score of each sample in the HALLMARK Pathway, and computed the correlation between JDP2 and HMOX1 and the score of each pathway, respectively. In JDP2, INTERFERON ALPHA RESPONSE, INTERFERON GAMMA RESPONSE, ALLOGRAFT REJECTION and COMPLEMENT are four pathways with significant positive correlation (Fig 6A). In HMOX1, REACTIVE OXYGEN SPECIES PATHWAY, IL2 STAT5 SIGNALING, PI3K AKT MTOR SIGNALING, and IL6 JAK STAT3 SIGNALING and COMPLEMENT are the four pathways with significant positive correlation (Fig 6B). Comprehensive analysis indicated that the two gene organisms had strong correlation with immune-related pathways.

**Fig 6:** The association of biomarkers with biological pathways. A: The correlation between JDP2 and pathway score; B: The correlation between HMOX1 and pathway score.

## 4 Discussion

PCOS is a common endocrine disorder in women [32]. Women with PCOS are often associated with a range of metabolic dysfunctions, including insulin resistance and obesity [33, 34]. Currently, more and more studies have demonstrated the identification of genes that characterize the pathogenesis of PCOS and help in the clinical diagnosis and treatment of PCOS. He et al. screened a total of seven important PCOS target genes based on the GEO database and weighted gene co-expression network analysis, including APOC3, ADCY2, C3AR1, HRH2, TAAR2, GRIA1, and MLNR [35]. The central gene OGN between PCOS and ovarian cancer was identified by bioinformatics by Zou et al. They showed that OGN regulates hormonal responses in PCOS and ovarian cancer, and found that OGN is strongly associated with desiccated iron anemia [36]. In this study, after multiple screening, we acquired two promising biomarkers JDP2 and HMOX1.Jun Dimerization Protein 2 (JDP2) is a member of the basic leucine zipper transcription factor family, and has diversified functions. It can be used as a cAMP response element and a histone chaperone to participate in and regulate important life processes. Such as cell cycle regulation, cell proliferation, cell apoptosis, can also be used as an oncogene to participate in the control of cell canceration [37]. Shimrit Avraham et al. found that JDP2 may also be involved in the regulation of SDF-1 expression in fibroblasts, a process that occurs frequently in tumor tissues and may inhibit the proliferation of cancer cells [38]. It has been found that CPG16 (a serine/threonine kinase) in pancreatic cells phosphorylates JDP2 by binding to it, reducing the activity of insulin promoters [39]. Notably, Jonak et al. showed that functional disruption of JDP2 can lead to early cessation of reproductive function and that this is associated with elevated follicle-stimulating hormone in women [40].

The article "Screening of potential biomarkers for polycystic ovary syndrome and identification of expression and immune characteristics" was retracted in 2025. Reasons: unreliable results or conclusions; concerns about the methods.

Heme Oxygenase-1 (HMOX1) can catalyze the degradation of heme, which produces carbon monoxide, iron bivalent ion and biliverdin to prevent ischemic injury and other diseases [41]. Overexpression of HMOX1 may increase the content of iron ions, resulting in ferroptosis of cardiomyocytes, and eventually induce cardiomyopathy [42]. HMOX1, found in another infertility disorder, endometriosis, may play a key role in embryonic ferroptosis, including stabilizing mitochondria to function properly to stop ferroptosis [43, 44]. Maowei Ni et al. found in ovarian cancer that co-treatment with Shikonin and cisplatin may increase HMOX1 expression levels and help induce ferroptosis in cancer cells [45]. It has also been found that high HMOX1 expression levels are associated with higher macrophage infiltration and lower mitochondrial complex levels [46].

PCOS can lead to complex immune system disorders characterized by chronic low-grade inflammation [47]. According to the results of GO and KEGG enrichment analysis and GSEA enrichment analysis of DEGs, we found that the enrichment degree of immune-related genes and pathways was high in PCOS. The scores of most immune cells and the degree of immune infiltration were significantly higher in the PCOS group. This can lead to severe immune and inflammatory reactions in patients. Inflammatory factors such as interleukin-1β released by relevant cells may play a pathological role in PCOS [48]. The biomarkers we screened, JDP2 and HMOX1, were highly correlated with immune-related pathways. JDP2 has been shown to be associated with the immune system in several studies. Pan et al. screened nine key genes (including JDP2) most associated with chronic lymphocytic leukemia by ferroptosis-based screening and constructed a risk model. They showed that the immune cell type and immune-related pathways of these patients were correlated with the risk score obtained from this model [49].

In this project, we screened potential biomarkers of PCOS, and identified the expression characteristics and immune characteristics of the biomarkers. The diagnostic ability and accuracy of biomarkers were verified by ROC curve and confusion matrix. We expect that our study will inform the development of clinical diagnosis and treatment strategies for PCOS.

There are still some limitations in this study. First of all, the pathological study on PCOS is still unclear, and we only chose GC expression profile data for analysis. However, the tissues and cells involved in PCOS are diversified, so comprehensive studies on the tissues involved in PCOS are still needed. Secondly, the experimental data came from the GEO database, and the sample size was insufficient. In the future, it is necessary to validate the role of our screened genes, including HMOX1 and JDP2, by performing further in vivo or in vitro validation experiments.

The article "Screening of potential biomarkers for polycystic ovary syndrome and identification of expression and immune characteristics" was retracted in 2025. Reasons: unreliable results or conclusions; concerns about the methods.

## 5 Conclusion

93 DEGs were identified in PCOS, and enrichment analysis revealed that the set of immune-related genes was differentially activated in PCOS. Recursive feature elimination (RFE) and LASSO regression were used for further feature selection of these genes, and finally JDP2 and HMOX1 were acquired as candidate biomarkers for PCOS.

## Supporting information

S1 Fig PCA analysis of JDP2 and HMOX1 distinguishing between PCOS and normal samples. JDP2 and HMOX1 could distinguish between PCOS (A) and normal (B) samples in both the training and validation cohorts.
(PDF)

S2 Fig Relationship between PCOS-related genes and immunomodulation-related genes. Relationship of PCOS-related genes to chemokine (A), immunoinhibitory (B), immunostimulatory (C), MHC (D) and receptor-related genes (E).
(PDF)

S1 Table Gene set of 28 immune cells. (CSV)

## Abbreviations

BP: biological process
CC: cellular component
DEGs: Differential Expressed Genes
GC: granulosa cell
GEO: Gene Expression Omnibus
GO: Gene Ontology
GSEA: Gene Set Enrichment Analysis
HMOX1: Heme Oxygenase-1
IR: insulin resistance
JDP2: Jun Dimerization Protein 2
KEGG: Kyoto Encyclopedia of Genes and Genomes
MF: molecular function
PCOS: polycystic ovary syndrome
RFE: Recursive feature elimination
ROC: Receiver Operating Characteristic
ssGSEA: Single sample gene set enrichment analysis
